The article "Prognostic Analysis of Elderly Patients with Multiple Organ Dysfunction Syndrome Undergoing Invasive Mechanical Ventilation" was published in 2020. Journal: J Healthc Eng.

# Prognostic Analysis of Elderly Patients with Multiple Organ Dysfunction Syndrome Undergoing Invasive Mechanical Ventilation

**DOI:** 10.1155/2020/6432048

**Published:** 2020-03-19

**Authors:** Kun Xiao, Bin Liu, Wei Guan, Peng Yan, Licheng Song, Yue Wang, Lixin Xie

**Affiliations:** ^1^Department of Pulmonary & Critical Care Medicine, Chinese People's Liberation Army (PLA) General Hospital, Beijing, China; ^2^Department of General Surgery, The 8th Medical Center of Chinese People's Liberation Army (PLA) General Hospital, Beijing, China

## Abstract

**Objective:**

To prospectively investigate early prognostic assessments of patients with Multiple Organ Dysfunction Syndrome in the Elderly (MODSE) who were receiving invasive mechanical ventilation (IMV).

**Methods:**

The clinical data of 351 patients were enrolled prospectively between January 2013 and January 2018. The Acute Physiology and Chronic Health Evaluation II (APACHE II), APACHE III, Simplified Acute Physiology Score (SAPS II), and Multiple Organ Dysfunction Score (MODS) were calculated. According to the outcome of 28-day, the patients were divided into survivors and nonsurvivors. Additionally, based on whether weaning could be implemented, all patients were divided into a successful-weaning group and a failure-to-wean group.

**Results:**

According to the prognosis, the areas under the receiver operating characteristic curve of the APACHE II, APACHE III, SAPS II, and MODS scoring systems were 0.837, 0.833, 0.784, and 0.860, respectively. MODS exhibited the highest sensitivity, whereas APACHE II showed the highest specificity, and successful weaning was conducive to ameliorating patients' prognosis. Multivariate logistic regression analyses revealed that underlying lung disease, plasma albumin, serum creatinine level, number of failing organs, and IMV duration were related to prognosis of weaning, with odds ratios (ORs) of 1.447, 0.820, 1.603, 2.374, and 3.105, respectively.

**Conclusions:**

The APACHE II, APACHE III, SAPS II, and MODS systems could perform excellent prognostic assessment for patients with Multiple Organ Dysfunction Syndrome in the elderly. Underlying lung disease, plasma albumin, serum creatinine, number of failing organs, and IMV duration were independent prognostic factors of weaning in MODSE patients with invasive mechanical ventilation.

## 1. Introduction

Invasive mechanical ventilation (IMV) is a life support measure that is widely applied in clinics and greatly improves the symptoms and prognosis of patients with respiratory failure, especially for those patients with Multiple Organ Dysfunction Syndrome in the Elderly (MODSE). However, previous study had demonstrated that long duration of IMV could lead to poor outcome [1] and would be an independent predictor of increasing hospital-mortality [2, 3] such as elderly patients undergoing IMV had an in-hospital mortality of 58% and a 6-month mortality of 67% [4, 5]. Thus, it is expected that MODSE patients undergoing IMV may have a poor prognosis, possibly due to the ventilator-associated lung injury and ventilator-associated inflammation [6]. Here, we attempted to perform early prognosis assessments for MODSE patients undergoing IMV using several scoring systems, including Acute Physiology and Chronic Health Evaluation II (APACHE II) [7] Acute Physiology, Age, Chronic Health Evaluation (APACHE III) [8] Simplified Acute Physiology Score (SAPS II) [9], and Multiple Organ Dysfunction Score (MODS) [10]. In addition, we also investigated the potential correlation factors of weaning for these patients.

The article "Prognostic Analysis of Elderly Patients with Multiple Organ Dysfunction Syndrome Undergoing Invasive Mechanical Ventilation" was published in 2020. Journal: J Healthc Eng.

## 2. Methods

### 2.1. Sample

This study enrolled 6512 patients, prospectively, who were treated in multiple ICUs of the General Hospital of the People's Liberation Army (PLA) and the 8th medical center of Chinese PLA General Hospital (including the Emergency Intensive Care Unit (EICU), the Surgical Intensive Care Unit (SICU), and the Medicine Intensive Care Unit (MICU)) between January 2013 and January 2018.

### 2.2. Inclusion and Exclusion Criteria

The inclusion criteria were as follows: (1) the patient was 60 years of age or older and met the multiple organ dysfunction definition proposed by Marshall et al. in 1995 [10]; (2) endotracheal intubation (via the nose or mouth) was implemented within 24 hours after admission to the ICU for invasive mechanical ventilation; and (3) the prognosis was well-defined. The exclusion criteria were the following: end stage of disease and exhibited multiple organ failure [10]; ICU stays of less than 24 h; invasive MV prior to entering the ICU; subjects had significant loss of clinical information and were as such difficult to score; and the patient, with an unknown prognosis, was discharged upon his or her request.

A total of 351 cases among 749 MODSE patients with complete clinical information were obtained and constituted the database of MODSE patients undergoing IMV, of which there were 327 cases of respiratory failure, 288 cases of heart failure, 245 cases of renal failure, 159 cases of liver failure, 74 cases of gastrointestinal dysfunction, 203 cases of neurological dysfunction, and 194 cases of coagulation disorders. Among the study subjects, there were 274 cases which were allowed to wean from MV, as they met the conditions for weaning, whereas 77 did not meet the standard during the ICU stay (Figure 1).

All participants signed an informed consent upon admission to the ICUs. This study was approved by the Clinical Ethics Committee of the General Hospital of the PLA.

The article "Prognostic Analysis of Elderly Patients with Multiple Organ Dysfunction Syndrome Undergoing Invasive Mechanical Ventilation" was published in 2020. Journal: J Healthc Eng.

### 2.3. Methods of the Prospective Study

Among the 749 enrolled MODSE patients, 351 patients who were undergoing IMV were analyzed prospectively. Many disease information should be collected, including the worst parameter among various vital signs (body temperature, heart rate, respiratory rate, blood pressure, urine volume, etc.), laboratory test results (blood routine, blood biochemistry, and coagulation parameters), and the clinical data (gender, age, ICU entry diagnosis, ICU stay duration, underlying disease). In addition, the APACHE II, APACHE III, SAPS II, and MODS results were calculated for the participants within 24 h after their ICU entry. Based on the outcomes upon ICU discharge, the participants were divided into a survival group and a nonsurvival group. Based on weaning criteria, the participants were divided into a weaning group (274 cases) and a nonweaning group (77 cases); depending on whether weaning would be successful, the weaning eligible individuals were further divided into a successful-weaning group (105 cases) and a failure-to-wean group (169 cases). If the datum for a parameter was missing, it was considered to be a default value of normal. ICU discharge (survival or death) was adopted as the observation end point. Multivariate logistic regression was performed to analyze individual parameters to identify the factors influencing weaning.

### 2.4. Evaluation Criteria

The weaning criteria previously reported [11] were employed herein: (i) adequate oxygen tension (under a condition of FIO_2_ 40% and positive end-expiratory pressure (PEEP) ≤5 cmH_2_O, blood oxygen saturation ≥90%); (ii) a stable cardiovascular system (heart rate ≤140 beats/min and stable blood pressure, without taking vasoactive drugs); (iii) sufficient consciousness, without continuously taking sedatives; (iv) normal body temperature (36–37.2°C); (v) satisfactory cough reflex during suctioning, with a gradually decreasing suctioning frequency; (vi) a lack of respiratory acidosis; and (vii) rapid shallow breathing index (tidal volume/respiratory frequency) ≤105.

The criteria of successful weaning included the following [12]: patients could be liberated from the endotracheal tube without requiring reintubation/MV for more than 48 hours after extubation, and so that the patient had stable vital signs and reported no obvious discomfort. The blood gas analysis revealed no respiratory acidosis exhibited no respiratory acidosis (blood gas analysis) and did not receive another intubation procedure.

The criteria of failed weaning were as follows: reintubation within 48 hours, a participant was considered to experience weaning failure if he/she died or needed to receive another procedure of MV.

The article "Prognostic Analysis of Elderly Patients with Multiple Organ Dysfunction Syndrome Undergoing Invasive Mechanical Ventilation" was published in 2020. Journal: J Healthc Eng.

### 2.5. Statistical Analyses

SPSS 17.0 software was employed herein for statistical analyses. Measurement data consistent with a normal distribution were all expressed as means ± standard deviations ($\bar{x}$ ± *s*); comparisons between two groups were facilitated by the *t* test. Skewed distribution data were expressed as medians; comparisons between two groups were facilitated by the Kruskal–Wallis rank sum test. Qualitative data, expressed as rates, were used to describe frequencies or intensities of occurrence and were examined using the *x*^2^ test. The receiver operating characteristic curve (ROC curve) was employed for determining the assessment performance of individual scoring systems, during which the sensitivity, specificity, and *Youden Index* of each prognosis score was calculated; the area under the curve (AUC) and the 95% confidence interval (95% CI) were obtained before significance tests were performed. Univariate and multivariate logistic regression analyses of dichotomous variables were performed to investigate prognosis-influencing factors for MODSE patients undergoing MV. *p* < 0.05 was considered statistically significant.

## 3. Results

### 3.1. General Information

Among the 749 enrolled MODSE patients from 6 ICU-centers, 351 (46.83%) were received IMV and had a mean age of 77.7 ± 9.2 years. Of the 351 patients, there were 254 males (72.46%) and 97 females (27.64%); there were 102 survivors (29.06%) and 249 nonsurvivors (70.94%) based on the outcome of 28-day; there were 274 individuals who met the ventilator weaning criteria (78.06%), including 105 cases (76 survivals and 29 deaths) of successful weaning (38.32% of the 274) and 169 cases (26 survivals and 143 deaths) of failed weaning (61.68% of the 274); and there were 64 participants undergoing tracheotomy (26 in the weaning failure subgroup, and 38 in the nonweaning group). These general statistics are summarized in Table 1.

### 3.2. Comparison of the Prognosis Assessments for MODSE Patients Undergoing MV

Based on the survival/death upon discharge (or ICU discharge), prognosis was assessed using the worst scores (APACHE II, APACHE III, SAPS II, and MODS) during the first 24 h of ICU entry, before the ROC curve was plotted. The score corresponding to the maximal Youden index was set as the optimal cutoff value, whereby the individual sensitivities, specificities, Youden indices, AUCs, and 95% confidence intervals were calculated (Table 2, Figure 2).

### 3.3. General Clinical Information of the Two Weaning Groups

Depending on the weaning outcome, the subjects were divided into a weaning success subgroup and a weaning failure subgroup. The prognostic differences of the two subgroups were evaluated (Table 3). This study indicated that successful weaning would help improve the prognosis of patients with mechanical ventilation.

The article "Prognostic Analysis of Elderly Patients with Multiple Organ Dysfunction Syndrome Undergoing Invasive Mechanical Ventilation" was published in 2020. Journal: J Healthc Eng.

### 3.4. Logistic Regression Analysis for MODSE Patients with IMV

Logistic regression analysis of dichotomous variables was performed to screen the factors influencing weaning. First, the 274 weaning-eligible patients were divided into a weaning success subgroup and a weaning failure subgroup. Their clinical data were subsequently documented, including their gender, age, number of organs with failure, concurrent diseases (e.g., hypertension, diabetes, chronic obstructive pulmonary disease, coronary heart disease, and immunosuppression), worst vital sign within 24 h of ICU entry, and laboratory test results. These parameters were then introduced into univariate and multivariate logistic regression equations of dichotomous variables. Underlying lung disease, plasma albumin, serum creatinine level, number of organs with failure, and IMV duration fit into the regression equation, indicating that the five parameters were independent factors influencing the weaning success rate for MODSE patients receiving IMV, with odds ratios (ORs) of 1.447, 0.820, 1.603, 2.374, and 3.105, respectively (Table 4).

## 4. Discussion

MODSE refers to conditions in which elderly individuals with multiple underlying diseases experience decreased organ function and reserve capacity. As a consequence, they are vulnerable to infections and display aggravated progression, leading to critical conditions that urgently require multiple organ support therapy (MOST). In this study, 53.97% of the MODSE patients underwent the life support treatment of IMV to alleviate symptoms and improve prognosis. However, long-term IMV may lead to ventilator dependence and difficulty in weaning, which elevates medical expenditure, decreases quality of life, and increases mortality.

Our data from multiple centers revealed that MODSE patients receiving IMV had poor prognosis and a high mortality rate of 71.07%. Comparison between the mortality group and the survival group revealed that the former had a slightly higher mean age, but the difference was not significant (*p*=0.816); gender was also not significantly different between the two groups. However, the mortality group had a significantly higher number of organs with failure (*p* < 0.001) and apparently poorer results for vital signs and laboratory results compared to the survival group. In addition, whether weaning was successful and whether reintubation was performed also had prominent influences on prognosis. The mortality group also had a significantly shorter ICU stay than the survival group, possibly because the mortality group had a higher number of organs with failure than the latter and correspondingly had more severe conditions. As a consequence, weaning failure compounded with reintubation might aggravate their disease and shorten their survival period [11, 13].

The article "Prognostic Analysis of Elderly Patients with Multiple Organ Dysfunction Syndrome Undergoing Invasive Mechanical Ventilation" was published in 2020. Journal: J Healthc Eng.

A scoring system consists of a set of objective quantitative indicators to evaluate disease severity and to assess prognosis. Its results indicate the degree of disease severity and the body's physiological dysfunction and can reliably reveal critical conditions and predict mortality risk [7–10]. Early determinations of disease severity and prognosis are crucial for clinical decision-making and allocation of ICU resources and are particularly important for MODSE cases with MV, who are characterized by a high mortality rate. Pettila et al. [14] conducted a prospective cohort study in which 520 MODS patients were evaluated to compare the predictive performances of four scoring systems, namely, APACHE II, MODS, Logistic Organ Dysfunction score (LODS), and Sequential Organ Failure Assessment score (SOFA). All four systems generated satisfactory performances in predicting patients' survival and death, with APACHE II showing the best performance for prognosis prediction. In this study, four scoring systems, namely, APACHE II, APACHE III, SAPS II, and MODS, were employed to perform early assessments for 351 MODSE patients undergoing IMV who had different prognosis. In comparison with the survival group, the in-hospital nonsurvival group exhibited significantly higher scores for APACHE II, APACHE III, SAPS II, and MODS (*p* < 0.05). The AUCs of the ROCs of these four scores were 0.837, 0.833, 0.784, and 0.860 and were not statistically significant. Among the four scoring systems, MODS performed the best sensitivity of 0.856, APACHE II produced the highest specificity of 0.835, and MODS showed the greatest AUC. The prognostic score markers are identical with not only in the population of old patients ICU. A single-center, retrospective cohort study of 905 patients showed that APACHE II score is also independently associated with the prognosis of patients given MV in the ICU among the patients from 17 to 98 years. Also, in the multivariate logistic regression analysis, APACHE II score was independently associated with higher odds of death in the patients aged <65 years [15]. Meanwhile, in our study, the APACHE II could perform excellent prognostic assessment for patients with Multiple Organ Dysfunction Syndrome in the elderly. These results indicated that MODS showed the best assessment performance and produced the highest sensitivity of prognosis assessment.

The article "Prognostic Analysis of Elderly Patients with Multiple Organ Dysfunction Syndrome Undergoing Invasive Mechanical Ventilation" was published in 2020. Journal: J Healthc Eng.

Early weaning and extubation followed by spontaneous breathing is the eventual goal of MV [16]. This study revealed that weaning outcome exhibited a significant influence on the patients' prognosis such that the weaning success subgroup exhibited an apparently superior prognosis to those of the weaning failure subgroup and the nonweaning group (*p* < 0.05). In this study, the weaning failure rate reached 61.69%, and the weaning failure subgroup exhibited significantly higher values in terms of mean age and number of organs with failure and a significantly shorter ICU stay compared with the weaning success subgroup (*p* < 0.05). These findings suggested that individuals who had relatively high age, who had underlying lung diseases, and whose conditions were compounded with multiple organ failure had increased disease severity and weaning risk and poor prognosis, in agreement with a previous study [17]. In the weaning success subgroup, 12% of the participants underwent tracheotomy, whereas in the weaning failure subgroup, 25% of the subjects had this procedure. It has been reported that early tracheotomy might decrease the possibility of complications such as pneumonia [18]. In addition, Griffiths et al. [19] revealed that early tracheotomy could shorten ICU stay but did not significantly affect mortality. In this study, the weaning failure subgroup exhibited a markedly higher mortality rate (81.05%) than that of the weaning success subgroup, which was consistent with a previous study [11]. It has been proposed that the high mortality and decreased extubation success rate in patients with failed weaning were related to the timing of reintubation [13].

To investigate the factors influencing weaning, multivariate logistic regression analyses of dichotomous variables were performed to identify indicators related to weaning success, which included underlying lung disease, plasma albumin, serum creatinine level, number of organs with failure, and MV duration, with ORs of 1.447, 0.820, 1.603, 2.374, and 3.105, respectively. As such, the data indicated that a high plasma albumin level is an independent protective factor for MODSE patients to wean from MV. In contrast, the other indicators (i.e., underlying lung disease, serum creatinine level, number of organs with failure, and MV duration) were risk factors affecting MODSE patients' weaning.

Plasma albumin can reliably reveal a patient's recent nutritional status. Under MV, the body is under stress conditions associated with robust energy consumption, metabolism, and decomposition activity, which can lead to relative malnutrition, manifested by a decreased plasma albumin level. In response, the body degrades respiratory muscle to compensate the energy deficit, which results in respiratory muscle atrophy and decreased muscle strength. Correspondingly, weaning from MV may cause respiratory muscle fatigue and, in turn, increase the risk of weaning failure [20]. In addition, the plasma albumin level is closely related to the prognosis of critical patients, especially elderly, hospitalized patients such that the lower the plasma albumin level is, the poorer are the nutritional status and the prognosis, and vice versa [21]. In other words, severe patients tend to be associated with an extraordinary weaning risk. In this study, we also revealed a pattern that the higher the number of organs with failure is, the higher is the severity scores (APACHE II and MODS). This finding indicated that critical patients are more likely to require various life support measures and have a relatively low likelihood of successful weaning. Serum creatinine level also influenced the prognosis of MODSE patients undergoing MV. Creatinine is an important indicator reflecting renal function. When the serum creatinine level reaches a uremic period, it can cause uremic lung or uremic pulmonary edema, in which alveoli exhibit diffusion dysfunction. As a consequence, pulmonary function is decreased, which causes weaning difficulty. Moreover, creatinine is also a catabolism product of muscle tissue in the body. Hence, an increased serum creatinine level indicates elevated body and muscle metabolism, which are not beneficial for the recovery and enhancement of respiratory muscle. Ultimately, weaning may cause respiratory muscle fatigue and decrease the possibility of weaning success.

The article "Prognostic Analysis of Elderly Patients with Multiple Organ Dysfunction Syndrome Undergoing Invasive Mechanical Ventilation" was published in 2020. Journal: J Healthc Eng.

In addition, it was reported that MV duration is also a crucial factor influencing whether weaning can be successful [22]. Protracted MV duration is associated with respiratory muscle structural damage and muscle fiber remodeling, which leads to ventilator dependency. Furthermore, long-term MV compromises the normal action of the diaphragm, which causes its dysfunction and reduces the weaning success rate.

## 5. Conclusions

In summary, the weaning of MODSE patients undergoing IMV is affected by complex and multisided factors. For these patients, it is important to actively provide impaired organs with functional support and to ameliorate or improve organ failure, thereby reducing the influences of intrapulmonary factors on weaning. In addition, it is also crucial to treat the primary disease, augment nutritional support, and improve the patient's condition. Among the critical scoring systems tested in this study, MODS exhibited the best performance of prognosis assessment for MODSE patients undergoing MV and is recommended for clinical application. Nevertheless, most indicators employed herein were extrapulmonary parameters, whereas intrapulmonary parameters, such as the rapid shallow breathing index [23], were not evaluated. As a consequence, the multivariate analyses may have generated biased conclusions.

## Figures and Tables

**Figure 1:** Flowchart of patient enrollment in this study.

**Figure 2:** The ROC curves for predicting prognosis of 28-day survivors and 28-day nonsurvivors.

**Table 1:** General clinical information of the enrolled patients.

	Total	28-day survivors (*n* = 102)	28-day nonsurvivors (*n* = 249)	*p*
Age (years)	77.71 ± 9.22	77.52 ± 9.18	77.86 ± 9.24	0.816
Gender (no., %)				
Male	254	72	182 (71.65%)	0.781
Female	97	30	67 (69.07%)	
Number of failing organs^*∗∗*^	3.82 ± 1.22	3.14 ± 1.03	4.09 ± 1.19	<0.001
Vital signs and laboratory tests				
Body temperature (°C)^*∗*^	37.81 ± 1.40	37.45 ± 1.25	37.95 ± 1.44	0.021
Heart rate (times/min)^*∗∗*^	114.7 ± 29.2	104.3 ± 26.1	118.9 ± 29.4	0.001
Breathing rate (times/minute)^*∗*^	24.5 ± 6.7	22.6 ± 5.6	25.3 ± 7.0	0.006
Mean arterial pressure (mmHg)	77.5 ± 22.6	82.1 ± 22.4	75.6 ± 22.5	0.070
Urine output (mL/24 hours)^*∗∗*^	1671.7 ± 1392.1	1371.8 ± 181.7	1332.1 ± 112.6	<0.001
WBC count (10^9^/L)^*∗*^	12.95 ± 8.20	11.19 ± 5.56	13.66 ± 8.98	0.021
Platelet count (10^9^/L)^*∗∗*^	126.5 ± 74.7	150.8 ± 69.3	116.7 ± 74.8	0.003
PaO_2_/FiO_2_^*∗∗*^	156.0 ± 85.0	180.7 ± 96.2	142.3 ± 76.2	<0.001
Serum creatinine (*μ*mol/L)^*∗∗*^	194.2 ± 173.0	141.5 ± 130.0	215.7 ± 183.7	0.002
Serum sodium (mmol/L)^*∗*^	140.05 ± 8.72	137.71 ± 7.01	141.00 ± 9.18	0.016
Serum potassium (mmol/L)^*∗∗*^	4.22 ± 1.10	3.78 ± 0.80	4.40 ± 1.16	<0.001
Serum albumin (g/L)	30.42 ± 8.72	32.32 ± 10.71	29.65 ± 7.68	0.050
Serum bilirubin (*μ*mol/L)^*∗∗*^	31.82 ± 61.00	16.43 ± 12.42	38.08 ± 71.05	0.001
Scoring systems				
APACHE II^*∗∗*^	25.6 ± 8.2	18.8 ± 6.1	28.4 ± 7.4	<0.001
APACHE III^*∗∗*^	96.5 ± 31.4	71.1 ± 24.6	106.9 ± 27.8	<0.001
SAPS II^*∗∗*^	61.9 ± 17.8	48.1 ± 13.3	67.6 ± 16.3	<0.001
MODS^*∗∗*^	8.7 ± 3.5	5.9 ± 2.5	9.9 ± 3.2	<0.001
Outcomes of weaning^*∗∗*^				
Success	105	76	29 (27.94%)	<0.001
Failure	169	26	143 (84.62%)	
The length of ICU stay (days)^*∗∗*^	20.93 ± 21.69	17.67 ± 19.99	28.95 ± 23.71	0.001

Quantitative data of normal distribution are presented as mean ± SD. Qualitative data are presented as *n*. ^*∗*^*p* < 0.05 and ^*∗∗*^*p* < 0.005 survivors *vs*. nonsurvivors. WBC counts: white blood cell counts. APACHE: Acute Physiology and Chronic Health Evaluation. SAPS: sample acute physiological score. MODS: multiple organ dysfunction syndrome. ICU: intensive care unit.

The article "Prognostic Analysis of Elderly Patients with Multiple Organ Dysfunction Syndrome Undergoing Invasive Mechanical Ventilation" was published in 2020. Journal: J Healthc Eng.

**Table 2:** Comparison of the diagnostic indicators of the prognostic scoring systems.

Scoring models	Cutoff	Se	Sp	Youden index	AUC	95% CI
APACHE II	25.5	0.769	0.856	0.604	0.837	0.768–0.898
APACHE III	86.0	0.748	0.809	0.557	0.833	0.752–0.890
SAPS II	57.5	0.698	0.762	0.420	0.784	0.706–0.832
MODS	6.5	0.816	0.827	0.643	0.860	0.797–0.916

Se: sensitivity; Sp: specificity; ROC curve: receiver operating characteristic curve; AUC: area under the curve; 95% CI: 95% confidence interval.

**Table 3:** Different prognostic outcomes of patients from different weaning groups/subgroups.

	Successful-weaning (*n* = 105)	Failure-to-wean (*n* = 169)	
Age (years)	76.5 ± 9.6	79.5 ± 8.8	0.050
Gender (no., %)			
Male	67	136	0.067
Female	38	33	
Underlying disease (no., %)			
Underlying lung disease^*∗∗*^	26	82	<0.001
Coronary heart disease	41	72	0.502
Hypertension	46	79	0.556
Diabetes	31	58	0.297
Number of failing organs^*∗∗*^	3.2 ± 1.0	3.9 ± 1.2	<0.001
Outcome of 28-day^*∗∗*^			0.001
Survivors	76	26	
Nonsurvivors	29	143	
The length of ICU stay (days)^*∗*^	19.4 ± 13.1	26.8 ± 24.4	0.034

^*∗*^ *p* < 0.05 and ^*∗∗*^*p* < 0.005 successful-weaning and failure-to-wean.

**Table 4:** Logistic regression analysis for MODSE patients with IMV.

Variable	B	Se	Wald	d*f*	*p* value	OR	95% CI
Underlying lung disease	0.439	0.156	6.796	1	0.001	1.447	1.098–1.816
Serum albumin	-0.085	0.033	5.890	1	0.021	0.820	0.732–0.924
Serum creatinine	0.004	0.003	2.913	1	0.036	1.603	1.210–1.974
Duration of MV	1.475	0.327	7.372	1	0.001	2.441	1.742–2.837
The number of failing organs	0.427	0.141	9.876	1	0.001	3.105	2.313–3.795

## Data Availability

The clinical data used to support the findings of this study have not been made available because of the protection of patient privacy.
